# Development and Validation of a Nomogram for Predicting Overall Survival to Concurrent Chemoradiotherapy in Patients with Locally Advanced Esophageal Squamous Cell Carcinoma

**DOI:** 10.1155/2022/6455555

**Published:** 2022-07-14

**Authors:** Chenyu Wang, Xinyu Cheng, Linzhi Jin, Runchuan Ren, Shaohua Wang, Anping Zheng, Anlin Hao, Fuyou Zhou, Yaowen Zhang

**Affiliations:** Department of Radiotherapy, Anyang Tumor Hospital, The Affiliated Anyang Tumor Hospital of Henan University of Science and Technology, Henan Medical Key Laboratory of Precise Prevention and Treatment of Esophageal Cancer, Anyang 455000, China

## Abstract

This study aims to develop and validate a effective prognostic nomogram for locally advanced esophageal squamous cell carcinoma (LA-ESCC) patients undergoing concurrent chemoradiotherapy (CCRT). Retrospective analysis of 503 patients with LA-ESCC given CCRT in our hospital from 2009 to 2016 was conducted. Two-thirds of the patients were randomly assigned to the training set (*n* = 335), and one-third were assigned to the validation set (*n* = 168). In order to generate the nomogram, multivariate cox regression analysis was undertaken in the training set for uncovering significant prognostic variables for overall survival. The *C*-index and calibration plot were used to verify nomogram discrimination and calibration, respectively. Five independent prognostic variables were found and incorporated into a nomogram: age, N stage, location, tumor response, and MLR (monocyte/lymphocyte ratio). The *C*-indexes of the training set and the validation set were 0.730 and 0.745, respectively. The discrimination and calibration of this nomogram showed good predictive power in both sets. Conclusively, the proposed nomogram may be served as an effective tool for prognostic evaluation of LA-ESCC patients receiving CCRT.

## 1. Introduction

Esophageal carcinoma is one of China's leading five malignant cancers, ranking third among newly diagnosed malignant tumors in males and fifth in females. The death rate of esophageal cancer ranks fourth among all malignant tumors [1]. Definitive concurrent chemoradiotherapy (CCRT) is the first choice for nonsurgical treatment of locally advanced esophageal carcinoma. However, the efficacy of CCRT varies substantially in these populations, with a five-year overall survival (OS) rate ranging from 20% to 44% [2, 3]. Although several clinicopathological factors are linked to survival and recurrence, it remains difficult to properly estimate the prognosis of locally advanced esophageal squamous cell carcinoma (LA-ESCC) patients receiving CCRT [4–7].

For clinicians to establish treatment plans and follow-up methods and to offer patients and their families meaningful information about short-term and long-term prognoses, accurate cancer prognostic prediction is vital. While the TNM staging system may be useful for predicting survival in general, the risk stratification system may not be suitable for evaluating the prognosis of specific individuals.

It is currently established that cancer survival is connected with the systemic inflammatory response [8, 9]. The communication between inflammatory and tumor cells is crucial in tumor microenvironment formation [10, 11]. Studies have shown that higher pre-treatment neutrophil/lymphocyte ratio (NLR), platelet/lymphocyte ratio (PLR), or monocyte/lymphocyte ratio (MLR) predicts a poorer prognosis in several cancer types [12–17].

Zhang et al. [6] reported utilizing nomogram to predict OS rate in LA-ESCC patients undergoing radiotherapy. Due to the fact that this nomogram was derived from LA-ESCC patients treated with radiotherapy alone or CCRT, its potential to predict OS in CCRT patients may be restricted. So far, no nomogram specifically predicting the OS rate of LA-ESCC patients receiving CCRT was reported. Therefore, the objective in this study was to develop and validate a nomogram based on inflammatory cells and clinicopathological characteristics to predict individual OS in LA-ESCC patients undergoing CCRT.

## 2. Methods

### 2.1. Patients

Patients with LA-ESCC who received initial CCRT treatments at Anyang Tumor Hospital between 1 January 2009 and 31 December 2016 were evaluated retrospectively. The following were the criteria for inclusion: (1) pathologically proven ESCC; (2) patients in clinical stages II-III were ineligible for surgery or declined surgery; (3) the dose of radiation was between 50 Gy and 70 Gy; (4) two cycles of cisplatin/fluorouracil (PF) or taxol/cisplatin (TP) chemotherapy were administered concurrently. Exclusion criteria: (1) history of infection within one month before therapy and (2) history of rheumatoid immunological disorders. Clinical staging was performed using the sixth edition of the TNM staging system of the American Joint Committee on Cancer (AJCC). This research was approved by the Anyang Tumor Hospital Ethics Committee. All patients provided informed consent in writing.

### 2.2. Data Collection

Age, gender, tumor length, location, TNM stage, radiotherapy dose, radiotherapy type, and adjuvant chemotherapy were gathered as demographic and clinicopathological data. Routine blood examinations were performed within one week before treatment to record the platelet, neutrophil, lymphocyte, and monocyte counts. The peripheral blood monocyte-, platelet-, and neutrophil-to-lymphocyte ratios (MLR, PLR, and NLR, respectively) were calculated.

### 2.3. Evaluation and Follow-Up

In order to evaluate the therapeutic outcome, esophagography, enhanced neck/thorax/abdomen CT scan, or PET-CT was conducted 4 weeks following the conclusion of CCRT. Tumor response was recorded as complete response (CR), partial response (PR), stable disease (SD), or progressive disease (PD) according to the revised solid tumor response assessment criteria guidelines (version 1.1) [18]. Follow-up began after patients receiving CCRT, through outpatient and inpatient case systems or telephone regular follow-up to understand the patient's condition. The most recent follow-up occurred on 31 December 2018. The primary outcome of interest was long-term OS.

### 2.4. Data Analysis

SPSS 26.0 (SPSS Inc., Chicago, IL, USA) and R software 4.0.2 (http://www.r-project.org/) with rms, survival, and survivalROC package were used for statistical analysis. A *P* < 0.05 was considered statistically significant in two-tailed statistical tests.

Two-thirds of the patients were allocated to the training set randomly, whereas one-third were allocated to the validation set to construct and verify the nomogram. Continuous variables were expressed as the means ± standard deviations, and categorical variables were expressed as a frequency or percentages. We observed that the MLR value was too small, so we multiplied it by 10 and labeled it per 0.1 change (henceforth MLR per 0.1 change). The chi-squared test or independent-samples *t*-test was carried out to compare the two sets of patients. The nomogram was constructed utilizing all important variables identified via a stepwise selection approach employing the Akaike information criterion (AIC) in multivariate Cox regression analysis of the training set [19]. To facilitate prediction of overall survival for individual patients, a straightforward and user-friendly website was created based on the nomogram (https://chenyuwang123.shinyapps.io/ospredict/).

Internal and external validations were conducted on the training and validation sets after developing the nomogram. Validation of the nomogram was determined by its ability to forecast individual outcomes (discrimination) and accurate estimations of the survival function point (calibration). Discrimination was measured using the concordance index (*C*-index) [20]. A *C*-index of 0.5 means no difference, while a *C*-index of 1.0 means that patients with different outcomes are completely separated. The calibration was assessed by calibration plots to illustrate the correlation between actual and predicted probabilities. Bootstrapping with 1,000 repeated samples was carried out for these activities to eliminate bias. According to the proposed nomogram, each patient's total points were determined for clinical application of this model. The optimal cutoff value was measured using the receiver operating characteristic (ROC) curve, and its accuracy was evaluated by the sensitivity and specificity. To further investigate the discriminative ability of the proposed nomogram, training set patients were separated into four groups by the quartiles of the nomogram total points, and the survival curve for each group was plotted. The Kaplan-Meier method was applied to generate the survival curves, and the log-rank test was conducted to determine the curve difference.

## 3. Results

### 3.1. Cohort Characteristics

A total of 503 patients were identified. In the training set (*n* = 335), the median follow-up was 34.3 months (range: 4.7 to 112.1 months). The median survival time (MST) was 36.2 months (95% CI: 29.9 to 49.6 months). The 3-year and 5-year OS rates were 50.2% and 38.1%, respectively. In the validation set (*n* = 168), the median follow-up was 35.6 months (range: 5.0 to 109.6 months). The MST was 36.2 months (95% CI: 28.2 to 55.6 months). The 3-year and 5-year OS rates were 49.8% and 36.1%, respectively. The clinical characteristics are reported in Table 1. Among all patients, males accounted for 65.4%, the mean patient age was 62.7 years old, 57.1% of the patients had lesions in the neck/upper thoracic esophagus, and 42.9% had lesions in the middle/lower thoracic esophagus. Nearly half of the patients had T4 (49.5%), whereas T1-T2 and T3 constituted 26.8% and 23.7%, respectively. 68% of patients were lymph node-positive, 24.5% were clinical stage II patients, and 75.5% were clinical stage III patients. With a mean radiation dose of 62.2 Gy, 56.7% of patients were given intensity-modulated radiotherapy (IMRT), and 43.3% received three-dimensional conformal radiotherapy (3DCRT). There were no significant differences in baseline data between training set and validation set.

### 3.2. Independent Prognostic Factors in the Training Set

Multivariate Cox regression analysis showed that age (*P* = 0.014), location (neck/upper vs. middle/lower, *P* < 0.001), N stage (N0 vs. N+, *P* < 0.001), tumor response (CR vs. PR, *P* < 0.001; CR vs. SD/PD, *P* < 0.001), and MLR (per 0.1 change) (*P* < 0.001) were linked to the OS independently (Table 2).

### 3.3. Prognostic Nomogram for OS

Figure 1 depicts the nomogram survival prediction for patients with LA-ESCC given CCRT. The nomogram relied on five independent prognostic variables: age, N stage, location, tumor response, and MLR (per 0.1 change). Based on the sum of the distribution points of each variable in the nomogram, a straight line could be drawn downward to measure the estimated 3- and 5-year survival probabilities.

### 3.4. Verification of the Nomogram

Predictions of the 3- and 5-year survival probabilities in the training and validation sets are depicted by the calibration curves shown in Figures 2 and 3, respectively. These calibration curves demonstrated excellent concordance between the predicted and observed 3- and 5-year OS rates. In the training set, the *C*-index was 0.730, and the corrected *C*-index was 0.724. In the validation set, the *C*-index was 0.745, and the corrected *C*-index was 0.746.  Table 3 lists the area under the ROC curve (AUC), an appropriate cutoff value of total nomogram points, and sensitivity and specificity for the prediction of 3- and 5-year survival probabilities. The training set patients were divided into four subgroups by quartiles of the nomogram total points to investigate the efficacy of the proposed nomogram in risk stratification, and the Kaplan-Meier curves were then plotted based on the nomogram-based groupings (Figure 4). The MST of each group (lowest to 81, 82 to 110, 111 to 138, and 139 to highest) was 82.7 months, 64.0 months, 23.9 months, and 19.3 months, respectively. The differences in survival time among subgroups were statistically significant (*P* < 0.001).

## 4. Discussion

The survival rates of patients with LA-ESCC administered CCRT vary greatly among individuals, and it is not accurate to evaluate the prognosis solely based on traditional staging systems. Although a nomogram of LA-ESCC patients receiving radiotherapy has been previously reported, one specifically for LA-ESCC patients undergoing CCRT has not been described. Hence, the prognostic nomogram for predicting the OS of this population was developed and verified in this study.

Five prognostic variables were identified in this study as being independently associated with the survival of patients with LA-ESCC, namely, age, tumor response, location, N stage, and MLR. Inflammation and innate immunity play important and complex roles in the development of various cancers. Inflammatory cells can change the tumor microenvironment through overproducing cytokines, including IL-2, IL-6, and TNF-*α*, thus promoting tumorigenesis and the proliferation, migration, and immune escape of tumor cells [21]. Meanwhile, immune cells are recruited and attenuate the inflammatory response to prevent cancer growth and progression. Some studies have suggested that poor survival rates are associated with a higher NLR in non-small-cell lung cancer, metastatic colorectal cancer, esophageal cancer, and advanced gastric cancer [14–17]. In contrast to the NLR, another study has found that PLR is an independent predictor of prognosis for esophageal cancer [13]. In addition, Basile et al. [12] have discovered that a high MLR indicates a poor prognosis of metastatic colon cancer patients. Moreover, Zhou et al. [22] have found that MLR is an independent prognostic factor of esophagogastric junction cancer patients, while NLR and PLR are not. In our study, the MLR was an independent predictor of the prognosis of LA-ESCC patients receiving CCRT. The inconsistency of various research results may be due to different baseline values of inflammatory cells, patients, or treatment methods.

As a prediction tool for cancer patients, MLR is supported by the following theory. First, tumors can recruit circulating monocytes and induce their differentiation into macrophages at the tumor site. Experiments have demonstrated that macrophages can accelerate tumor migration and metastasis by promoting angiogenesis in tumor tissue [23]. In contrast, lymphocytosis is more prevalent in cancer patients. Moreover, lymphocytes play a crucial part in the antitumor immunity of the host by enabling the death of cytotoxic cells, thus suppressing tumor cell proliferation and metastasis [24]. The MLR reflects the complex interaction between monocytes and lymphocytes in the tumor microenvironment as well as the equilibrium between the inflammatory and immunological responses of the host.

In addition to MLR, tumor response was also an independent prognostic factor for LA-ESCC patients who received CCRT in this study. The preoperative treatment response, notably the lack of residual disease in surgical specimens, has been consistently found in many studies to be an indication of improved disease-free survival and OS [25–27]. In a comprehensive review of esophageal cancer patients undergoing esophagectomy after neoadjuvant chemoradiotherapy, the survival rates were 2-3 times higher in patients with a pathological CR than in patients with residual disease in esophagectomy specimens [28]. Although the patients in our study did not undergo surgery, a clinical CR also indicated a higher possibility of a pathological CR. Similarly, Zhou et al. [7] and Zhang et al. [29] have reported that for patients with ESCC administered CCRT, a clinical CR is an independent predictor of the patient prognosis.

Our study suggested that the tumor location of middle/lower thoracic esophagus was a poor prognostic factor for LA-ESCC patients given CCRT. It is unclear why this is the case. We speculated that it might be caused by the high range of motion in the middle and lower esophagus during radiotherapy.

Besides the above factors, age and the N stage were also associated with the prognosis of LA-ESCC patients receiving CCRT. Most previous studies [4–6] have demonstrated the prognostic role of these factors in this population, and the observations in this study were in agreement with these previous findings.

Nevertheless, this study had some limitations. First, we divided patients into two groupings by chance. Two-thirds of the cases were utilized to build the nomogram, while the remainder were employed to validate it. Although this is a well-established approach when external cohorts are unavailable, this proposed nomogram must be verified in an external cohort-derived population. Second, the nomogram did not incorporate all potential predictors; therefore, it cannot make predictions with absolute precision. However, our results show that the nomogram based on five variables has good adaptability. Third, the proposed nomogram is based on ESCC, but increasing evidence indicates that squamous cell carcinoma and adenocarcinoma differ in etiology, epidemiology, tumor biology, and prognosis. Therefore, further research is required to determine if the proposed nomogram can be used for adenocarcinoma.

In conclusion, independent factors affecting the survival of LA-ESCC patients receiving CCRT were selected to develop a nomogram. The proposed nomogram may serve as an effective tool for prognostic evaluation of this population.

## Figures and Tables

**Figure 1:** Nomogram predicting survival in patients with locally advanced esophageal squamous cell carcinoma receiving concurrent chemoradiotherapy.

**Figure 2:** The calibration curve for predicting patient survival at (a) 3 years and (b) 5 years in the training set.

**Figure 3:** The calibration curve for predicting patient survival at (a) 3 years and (b) 5 years in the validation set.

**Figure 4:** Kaplan–Meier survival curves for patients stratified based on the quartiles of proposed nomogram total points in the training set.

**Table 1:** Characteristics of patients.

Variable	Total (*n* = 503)	Training set (*n* = 335)	Validation set (*n* = 168)	*P* value
Age (years, mean ± sd)	62.7 ± 8.4	62.5 ± 8.9	63.0 ± 7.2	0.594
Tumor length (cm, mean ± sd)	5.2 ± 2.1	5.2 ± 2.0	5.4 ± 2.3	0.357
Radiotherapy dose (Gy, mean ± sd)	62.2 ± 3.4	62.2 ± 3.4	62.2 ± 3.3	0.790
NLR (mean ± sd)	2.5 ± 1.5	2.5 ± 1.6	2.4 ± 1.1	0.468
PLR (mean ± sd)	144.5 ± 64.1	148.3 ± 68.2	136.9 ± 54.4	0.059
MLR (per 0.1 change) (mean ± sd)	0.3 ± 0.1	0.3 ± 0.1	0.3 ± 0.1	0.819
Sex (*n*, %)				0.674
Female	174 (34.6)	118 (35.2)	56 (33.3)	
Male	329 (65.4)	217 (64.8)	112 (66.7)	
Location (*n*, %)				0.429
Neck/upper	287 (57.1)	187 (55.8)	100 (59.5)	
Middle/lower	216 (42.9)	148 (44.2)	68 (40.5)	
T stage (*n*, %)				0.278
T1-T2	135 (26.8)	90 (26.9)	45 (26.8)	
T3	119 (23.7)	86 (25.7)	33 (19.6)	
T4	249 (49.5)	159 (47.5)	90 (53.6)	
N stage (*n*, %)				0.963
N0	161 (32.0)	107 (31.9)	54 (32.1)	
N+	342 (68.0)	228 (68.1)	114 (67.9)	
Clinical stage (*n*, %)				0.369
II	123 (24.5)	86 (25.7)	37 (22.0)	
III	380 (75.5)	249 (74.3)	131 (78.0)	
Radiotherapy type (*n*, %)				0.971
IMRT	285 (56.7)	190 (56.7)	95 (56.5)	
3DCRT	218 (43.3)	145 (43.3)	73 (43.5)	
Adjuvant chemotherapy (*n*, %)				0.469
No	267 (53.1)	174 (51.9)	93 (55.4)	
Yes	236 (46.9)	161 (48.1)	75 (44.6)	
Tumor response (*n*, %)				0.517
CR	113 (22.5)	78 (23.3)	35 (20.8)	
PR	351 (69.8)	234 (69.9)	117 (69.6)	
SD/PD	39 (7.8)	23 (6.9)	16 (9.5)	

NLR: neutrophil/lymphocyte ratio; PLR: platelet/lymphocyte ratio; MLR: monocyte/lymphocyte ratio; CR: complete response; PR: partial response; SD: stable disease; PD: progressive disease; IMRT: intensity-modulated radiotherapy; 3DCRT: three-dimensional conformal radiotherapy.

**Table 2:** Multivariate Cox regression of the training set.

Variable	*β*	HR	HR 95% CI	*Z* value	*P* value
Age	0.02	1.02	1.00-1.03	2.45	0.014
Location					
Neck/upper	1 [reference]	1 [reference]	1 [reference]	—	—
Middle/lower	0.64	1.90	1.45-2.49	4.64	<0.001
N stage					
N0	1 [reference]	1 [reference]	1 [reference]	—	—
N+	0.91	2.48	1.77-3.47	5.31	<0.001
Tumor response					
CR	1 [reference]	1 [reference]	1 [reference]	—	—
PR	0.85	2.34	1.61-3.40	4.47	<0.001
SD/PD	1.82	6.14	3.47-10.89	6.22	<0.001
MLR (per 0.1 change)	0.21	1.24	1.15-1.34	5.38	<0.001

HR: hazard ratio; CI: confidence interval; MLR: monocyte/lymphocyte ratio; CR: complete response; PR: partial response; SD: stable disease; PD: progressive disease.

**Table 3:** Accuracy of the proposed nomogram for predicting 3-year and 5-year survival probability.

Variable	Training set		Validation set	
	3 years	5 years	3 years	5 years
AUC	0.816	0.811	0.825	0.813
Cutoff point	116	111	115	114
Sensitivity (%)	72.8	70.3	74.4	65.3
Specificity (%)	81.0	84.9	79.0	85.0

AUC: area under the receiver operating characteristic curve.

## Data Availability

All the underlying data supporting the results of our study are in the manuscript.
